The article "Acute psilocybin increased cortical activities in rats" was retracted in 2026. Reasons: errors in the materials; unreliable results or conclusions.

# Acute psilocybin increased cortical activities in rats

**DOI:** 10.3389/fnins.2023.1168911

**Published:** 2023-05-23

**Authors:** Junhong Liu, Yuanyuan Wang, Ke Xia, Jinfeng Wu, Danhao Zheng, Aoling Cai, Haitao Yan, Ruibin Su

**Affiliations:** ^1^State Key Laboratory of Toxicology and Medical Countermeasures, Beijing Key Laboratory of Neuropsychopharmacology, Beijing Institute of Pharmacology and Toxicology, Beijing, China; ^2^Nanjing University of Chinese Medicine, Nanjing, China; ^3^State Key Laboratory of Magnetic Resonance and Atomic and Molecular Physics, Key Laboratory of Magnetic Resonance in Biological Systems, Wuhan Center for Magnetic Resonance, Wuhan Institute of Physics and Mathematics, Innovation Academy for Precision Measurement Science and Technology, Chinese Academy of Sciences, Wuhan, Hubei, China; ^4^The Affiliated Changzhou Second People's Hospital of Nanjing Medical University, Changzhou Second People's Hospital, Changzhou Medical Center, Nanjing Medical University, Changzhou, China

**Keywords:** psychedelics, psilocybin, fMRI, 5-HT2A, BOLD, EGR1 (early growth response protein 1), depression, functional connectivity (FC)

## Abstract

Psilocybin, a naturally occurring hallucinogenic component of magic mushrooms, has significant psychoactive effects in both humans and rodents. But the underlying mechanisms are not fully understood. Blood-oxygenation level-dependent (BOLD) functional magnetic resonance imaging (fMRI) is a useful tool in many preclinical and clinical trials to investigate psilocybin-induced changes of brain activity and functional connectivity (FC) due to its noninvasive nature and widespread availability. However, fMRI effects of psilocybin on rats have not been carefully investigated. This study aimed to explore how psilocybin affects resting-state brain activity and FC, through a combination of BOLD fMRI and immunofluorescence (IF) of EGR1, an immediate early gene (IEG) closely related to depressive symptoms. Ten minutes after psilocybin hydrochloride injection (2.0 mg/kg, i.p.), positive brain activities were observed in the frontal, temporal, and parietal cortex (including the cingulate cortex and retrosplenial cortex), hippocampus, and striatum. And a region-of-interest (ROI) -wise FC analysis matrix suggested increased interconnectivity of several regions, such as the cingulate cortex, dorsal striatum, prelimbic, and limbic regions. Further seed-based analyses revealed increased FC of cingulate cortex within the cortical and striatal areas. Consistently, acute psilocybin increased the EGR1 level throughout the brain, indicating a consistent activation thought the cortical and striatal areas. In conclusion, the psilocybin-induced hyperactive state of rats is congruent to that of humans, and may be responsible for its pharmacological effects.

The article "Acute psilocybin increased cortical activities in rats" was retracted in 2026. Reasons: errors in the materials; unreliable results or conclusions.

## 1. Introduction

Psilocybin, the prodrug of psilocin and a chemical analog of the neurotransmitter serotonin (5-HT), is a naturally occurring hallucinogenic component derived from magic mushrooms. Similar to other psychedelics, like lysergic acid diethylamide (LSD) and ayahuasca, psilocybin can induce hallucination in humans, and shows great therapeutic potential to several psychiatric disorders like depression and anxiety, which acts through, at least partially, activation of the brain’s serotonin system (Moreno et al., 2006; Thomas et al., 2017; Preller et al., 2020; Vollenweider and Preller, 2020; Daws et al., 2022). Binding studies suggest its high affinity for most serotonin receptors, including serotonin 5-HT_1A_ and 5-HT_2A_ receptors (NIMH Psychoactive Drug Screening Program database: https://pdsp.unc.edu/databases/pdsp.php), which are both important targets to psychiatric disorders therapy and are considered to constitute a bipartite model to modulate brain serotonin function (Carhart-Harris and Nutt, 2017).

Functional magnetic resonance imaging (fMRI) is becoming increasingly popular in basic research and drug development. Its non-invasive nature, good cross-species consistency, widespread availability, and unparalleled brain-wide spatial and temporal resolution render it a representative platform for translational and reverse-translational studies across humans and rodents (Lu et al., 2012; Sumiyoshi et al., 2019). In the past few decades, with the advancements of hardware apparatus and data processing methodologies, a plethora of studies have explored brain activity changes induced by psychiatric disorders and the chemical intervention using fMRI technique (Carhart-Harris et al., 2016; Müller et al., 2018; Roseman et al., 2018; Zheng et al., 2018; Daws et al., 2022). And the effects of psilocybin and other psychedelics (such as LSD and ayahuasca) on brain activity and functional connectivity (FC) in humans were investigated from different perspectives (see the review for detail (McCulloch et al., 2022)), among which altered activity was mostly reported in such “hub regions” as the anterior cingulate cortex (ACC), posterior cingulate cortex (PCC), medial prefrontal cortex (mPFC), and thalamus. Increased FC between ACC and PCC was observed after psilocybin treatment in major depressive patients (Doss et al., 2021), and optogenetic activation of mice mPFC also had antidepressive effects (Covington et al., 2010). It seems these ‘hub regions’ are crucial for psilocybin’s depression-relieving effects in humans and mice. Likewise, the rat cingulate cortex is fairly significant for interhemispheric communications despite some structural differences (Vogt and Paxinos, 2014). However, whether the cingulate regions in rats are crucial targets on psilocybin-induced brain activity changes has not been fully elucidated as of yet. Therefore, we hypothesized that these hub regions, like the cingulate cortex, may be the key regions affected by psilocybin in rats.

The article "Acute psilocybin increased cortical activities in rats" was retracted in 2026. Reasons: errors in the materials; unreliable results or conclusions.

When it comes to those important fMRI studies in humans, limitations still exist. For example, fMRI readouts are, in essence, an indirect reflection of neural mass activity, which are subject to both physical and biological constraints (Logothetis, 2008). And with the burgeoning of varied methodologies, diverse research may, sometimes, lead to differential results with the same data. Multifarious experimental designs and methodological techniques also bear additional difficulties in direct comparisons among different fMRI studies. What’s more, in human studies, it is not easy to directly compare the fMRI readouts with the postmortem molecular expression, even though this can be easily done in animals (Sumiyoshi et al., 2019).

Different from the indirect reflective nature of fMRI, immediate early genes (IEG) in the brain are critical mediators and direct indicators of neuron activity. These IEG are involved in various processes such as learning, memory, neuroplasticity, neural reaction to various stimuli, and psychiatric disorders (González-Maeso et al., 2007; Pérez-Cadahía et al., 2011; Leal et al., 2014; Minatohara et al., 2016; Chandra and Lobo, 2017; Duclot and Kabbaj, 2017; Jefsen et al., 2021). IEG *early growth factor 1* (*egr1*), a member of the *egr* family (Beckmann and Wilce, 1997), is widely expressed throughout the brain (Knapska and Kaczmarek, 2004) and its translational product, EGR1 protein (EGR1), is evolutionarily conserved across humans, mice, and rats (Poirier et al., 2008). More importantly, EGR1 levels are closely correlated with depression, anxiety, and schizophrenia (Duclot and Kabbaj, 2017). EGR1 level in mPFC was reported to be directly associated with the depression phenotype (Covington et al., 2010), and was even recommended as a marker of positive responses to antidepressant treatment (Minatohara et al., 2016). In patients with schizophrenia, decreased *egr1* mRNA levels in the dorsolateral prefrontal cortex (dlPFC) was observed, whereas there was an increase in fibroblasts and whole blood samples, the latter of which was associated with delusion states of schizophrenia patients (Yamada et al., 2007; Kurian et al., 2011; Cattane et al., 2015). Another study reported *egr1* as a biomarker specifically responsive to hallucinogenic 5-HT_2A_ receptor agonists relative to the non-hallucinogenic ones, in that psilocin, the active metabolite of psilocybin, significantly increased brain *egr1* mRNA level in normal mice but not in 5-HT_2A_ receptor knockout mice (htr2a^−/−^), suggesting the prerequisite role of 5-HT_2A_ receptor in the *egr1* induction in this context (González-Maeso et al., 2007). Therefore, EGR1 can be seen as a direct and specific indicator of neural activity induced by psilocybin.

The article "Acute psilocybin increased cortical activities in rats" was retracted in 2026. Reasons: errors in the materials; unreliable results or conclusions.

Given the noninvasive but indirect nature of fMRI and invasive but direct properties of IF in reflecting neural activities, we therefore combined BOLD fMRI and IF of EGR1, for the first time, to further investigate the effects of psilocybin on rat brain activity.

## 2. Materials and methods

### 2.1. Animals

A total of 91 male Sprague Dawley (SD) rats (Beijing HFK Bioscience Co. Ltd.), aged 7–9 weeks, weighing 230–260 g, were housed two or three per cage with food and water access *ad libitum*, under a 12 h: 12 h light/dark cycle (light on at 7: 00 a.m.), in a temperature- and humidity-controlled room (25 ± 2°C and 60% ± 10%, respectively). They were allowed to acclimatize to the environment for at least 1 week before experiments. In consideration of the enduring anesthetic effects of isoflurane on protein expression (Bunting et al., 2015) and long-term antidepressive effects of psilocybin (Thomas et al., 2017; Daws et al., 2022), all rats were used only once, of which 75 rats were used for head twitch response (HTR), 10 for fMRI scanning, and 6 for EGR1 IF. All experiments were carried out in accordance with the National Institute of Health Guidelines for the Care and Use of Laboratory Animals. Every effort was made to minimize discomfort to the animals.

### 2.2. Drugs and agents

Psilocybin hydrochloride (synthesized by the Beijing Institute of Pharmacology and Toxicology) was dissolved in 0.9% sterile saline solution with a final concentration of 0.2, 0.5, 1.0, and 2.0 mg/mL for the HTR experiment. The final dosage of 2.0 mg/kg psilocybin hydrochloride in fMRI and IF experiments was selected in reference to previous research (González-Maeso et al., 2007; Grandjean et al., 2021). For each experiment, psilocybin was dissolved immediately before the experiment and stored in a dark environment.

### 2.3. Head twitch response

Before the HTR experiment, each rat was acclimatized to a new housing cage alone with fresh padding material for 20 min to alleviate manipulation- and environment-induced stress. Next, rats were intraperitoneally (i.p.) administered with saline or psilocybin hydrochloride (2.0 mg/kg) in a volume of 0.1 mL/100 g body weight. After that, the animals were placed back in the cage immediately and the HTR within 30 min were manually counted by three experimenters who were blind to the treated agents.

The article "Acute psilocybin increased cortical activities in rats" was retracted in 2026. Reasons: errors in the materials; unreliable results or conclusions.

### 2.4. Immunofluorescence

Sixty minutes after treatment, the rats were deeply anaesthetized with sodium pentobarbital solution. Transcardial perfusion was then performed with 4% paraformaldehyde solution (PFA, Beijing Applygen Technologies Inc., China) and then with 0.1 M phosphate buffer (PBS) (Beijing Applygen Technologies Inc., China) for 10 min, respectively. The perfused brains were removed and saved in 4% PFA overnight and then dehydrated in 30% sucrose solution for 3–5 days. The dehydrated brain was frozen and sectioned into slices (30 μm thick) with a sliding microtome (RWD life science Co. Ltd., China) in the frontal plane and every one of six slices was selected as a series. The series was carefully washed and incubated with blocking buffer (Beyotime, China) for 2 h at 20°C, then with anti-EGR1 primary rabbit antibody (1: 1000, Cell Signaling Technology, United States, 44D5) for 10 h. The incubated slices were washed with 0.1 M PBS followed by anti-rabbit secondary antibody (1: 500, Cell Signaling Technology, United States, 4412S) immunostaining for 2 h at 20°C. After washing, the slices were counterstained and cover slipped using DAPI-containing mounting medium (Sigma-Aldrich, United States). The immunostained slices were fluorescently imaged using a slice scanner (Olympus VS200, Japan). Finally, the IF images were processed with ImageJ (National Institute of Health, USA) in reference to the stereotaxic rat atlas (Paxinos and Watson, 2007).

### 2.5. MRI scanning

MRI experiments were conducted using a Bruker Biospec70/20USR small animal MR system (Bruker, Germany) operating at 300 MHz (7 T). A partial volume transmit coil was used for signal transmission and a 10 mm surface coil for signal reception (Bruker, Germany). Before scanning, rats were anesthetized with 4% isoflurane (RWD life science Co. Ltd., China) and underwent abdominal catheterization using a homemade drug injection device. Those animals were carefully transferred to the animal bed of the MRI scanner, and their heads were fixed with two ear bars and a tooth bar. Isoflurane was gradually reduced to 2–3% to maintain the animals in a stable state with a steady respiration rate ranging between 60 and 80 breaths per minute. In addition, a homemade hot water circulation device was used to keep the animal’s body temperature constant.

During scanning, a 3D-FLASH and a Fieldmap image were collected for head location and preparation for the phase field correction. Then, repeated fieldmap correction and tuning were performed to improve the image quality. fMRI data were collected before and 10 min after drug injection. In detail, resting-state fMRI data were acquired using gradient echo EPI (GE-EPI) sequence with the following parameters: field of view (FOV) = 21.0 × 28.0 mm^2^, matrix size = 80 × 60, repetition time (TR) = 2000 ms, echo time (TE) = 14 ms, number of averages (NA) = 1, number of repetition (NR) = 300, spatial resolution = 0.35 × 0.35 mm^2^, slice thickness = 0.8 mm, slices number = 22 (no gap), and scan time = 10 min. A structure image was acquired at the same geometry using T2-weighted fast spin-echo sequence Turbo-RARE: FOV = 21.0 × 28.0 mm^2^, matrix size = 256 × 256, TR = 3,000 ms, TE = 12 ms, NA = 4, NR = 1, spatial resolution = 0.08 × 0.11 mm^2^, slice thickness = 0.8 mm, and slices number = 22 (no gap).

The article "Acute psilocybin increased cortical activities in rats" was retracted in 2026. Reasons: errors in the materials; unreliable results or conclusions.

### 2.6. MRI data analysis

All fMRI data was preprocessed with afni,^1^ fsl,^2^ ANTs,^3^ and homemade MATLAB code. The MRI data was first converted to NIFITI format using <Bru2Anz converter>.^4^ Then, the image orientation and image center were corrected using <3drefit>. The tissue outside of the brain was removed using <antsRegistrationSyN> and a homemade rat brain mask. The first five volumes were removed and slicetiming was performed using <3dTshift>. Head motion correction were performed using <antsMotionCorr> and 0.01–0.1 Hz temporal filter was performed using <3dBandpass>. For spatial correction, every EPI image was first rigid-body transformed to match their own T2-weighted images, and then nonlinear transformed to match a rat standard template (Sigma Wistar Rat Brain Template; Barrière et al., 2019) using <antsRegistrationSyN>. Finally, all the EPI images were smoothed using a FWHM of 0.3 mm^3^.

For degree centrality (DC) analysis, the correlation strengths between each voxel and every other voxel in the brain were calculated and a threshold of 0.2 (Liu et al., 2015) was used to exclude random connection. Finally, the degree centrality maps (weighted) were taken into statistical analysis. The difference image was obtained between before- and after-psilocybin injection using a voxel by voxel two-sample test; *p* < 0.05 was seen as statistically significant.

For ROI-wise functional connectivity analysis, in total 59 ROIs (Supplementary Table S1) were used according to the rat Sigma function brain atlas (Barrière et al., 2019). In the templates, the functional cingulate cortex was subdivided into Cg1, Cg2, and Cg3 (Supplementary Figure S1A). The average time courses of the 59 ROIs were extracted and the correlation strengths between each of them were calculated. Fisher-z transformation was performed on the correlation matrixes and the difference ROI-ROI pairs between before- and after-psilocybin were acquired using paired-sample test. To display the significantly changed ROI-ROI pairs in ROI-wise FC analysis, a threshold of *p* < 0.05 was used for the statistical analysis.

The article "Acute psilocybin increased cortical activities in rats" was retracted in 2026. Reasons: errors in the materials; unreliable results or conclusions.

For voxel-wise (seed-based) functional connectivity analysis, anatomical cingulate cortex (Supplementary Figure S1B) was chosen as the ROI and their average time course was extracted. All the correlation strengths between the time courses of voxels in the brain and the ROI time course were calculated. Fisher-z transformation was performed on the correlation maps and the difference images between before- and after-psilocybin were acquired using a voxel by voxel two-sample test; *p* < 0.05 was seen as statistically significant.

## 3. Results

### 3.1. Mixed pattern of BOLD signals after acute psilocybin treatment

First, to investigate how psilocybin affect rat brain activities, whole-brain resting state fMRI was performed and the degree centrality was analyzed before versus after a single dose of 2.0 mg/kg psilocybin hydrochloride. And a mixed pattern of brain activity alteration was presented (Figure 1), characterized by increased degree centrality in the cingulate cortex, prefrontal cortex (PFC), motor cortex, somatosensory cortex, insular cortex, dorsal striatum, hippocampus, and the superior part of some septal and thalamic areas, and by decreased degree centrality in the ventral striatum, inferior part of septum, basal thalamic nuclei, and some hypothalamic areas. Psilocybin produced a mixed pattern of brain activity changes in rats, which shows some similarity to its acute effects in human (Preller et al., 2020).

**Figure 1:** Psilocybin produced a mixed pattern of degree centrality (DC). Increased DC (red) was widespread in cortical, striatal, and hippocampal regions and decreased in subcortical regions. A threshold of 0.2 was used to exclude random connection, DC was analyzed using a two-sample test, and *p* < 0.05 was seen as statistically significant. Each positive (or negative) numerical value over brain sections is the AP value in the rat stereotaxic atlas, representing the distance anterior (or posterior) to bregma.

### 3.2. FC between cingulate cortex and other regions changed most

Subsequently, ROI-wise FC analysis was performed to investigate the interconnection changes across the whole brain for further analysis. The analysis matrix revealed that a great proportion of the affected regions showed increased FC with multiple regions, like the cingulate cortex, dorsal and ventral striatum, prelimbic/infralimbic areas, piriform cortex, primary somatosensory cortex, motor cortex, and ventral thalamic nucleus, among which the FC of the cingulate cortex changed the most (Figure 2). Regions showing decreased FC with others were the insular cortex, accumbens shell, retrosplenial granular area, and parietal (auditory) cortex. And the FC of retrosplenial granular cortex showed the most decrement of these. Moreover, a bilateral fluctuation of FC changes was observed in the insular cortex and piriform cortex. Considering the possibility that multiple comparison correction might cover the potential positive results, no multiple comparison correction was performed in this exploratory analysis. In general, the exploratory ROI-wise FC analysis abovementioned suggested the FC of several rat cingulate subregions like the cingulate cortex 1 (Cg1), cingulate cortex 3 (Cg3), homologous to the respective ACC and MCC of humans and crucial for inter-hemispheric communication (Vogt and Paxinos, 2014) with other brain regions, were intensively changed.

The article "Acute psilocybin increased cortical activities in rats" was retracted in 2026. Reasons: errors in the materials; unreliable results or conclusions.

**Figure 2:** Psilocybin changed brain functional connectivity. The rat brain was divided into 59 ROIs, FC between each ROI was analyzed using paired-sample t test without multiple correction, a threshold of *p* < 0.05 was used for the statistical analysis. White dots indicate increased FC between the two ROIs and black dots indicate decreased FC between them. Among the matrix, the FC of Cg (Cg1,3) and striatum changed most.

### 3.3. Bidirectional FC changes of cingulate cortex with several cortical and subcortical regions

After identifying the functional cingulate cortex as a core region according to rat Sigma function brain atlas (Barrière et al., 2019), in order to further verify the key role of the cingulate cortex in psilocybin-induced rat brain FC changes in a more precise way, seed-based FC analysis was performed using anatomical cingulate cortex (Paxinos and Watson, 2007) as the seed (Supplementary Figure S1B). Psilocybin was observed to increase rat cingulate connectivity with the olfactory bulb, orbital frontal cortex, anterior insular cortex, lateral part of somatosensory cortex, posterior entorhinal cortex, visual cortex, retrosplenial cortex, striatum, thalamus, hippocampus, postsubiculum, and periaqueductal grey, and decreased cingulate connectivity with the preoptic area, inferior part of septum, piriform cortex, amygdala, inferior thalamic areas, and substantia nigra (Figure 3).

**Figure 3:** Psilocybin-induced changes in Cg functional connectivity. Regions where activity show a positive coupling with Cg are shown in red, and negative in blue. Two-sample test was used and *p* < 0.05 was seen as statistically significant. Each positive (or negative) numerical value over the brain section is the AP value in the rat stereotaxic atlas, representing the distance anterior (or posterior) to bregma section.

The article "Acute psilocybin increased cortical activities in rats" was retracted in 2026. Reasons: errors in the materials; unreliable results or conclusions.

### 3.4. Psilocybin increased EGR1 expression throughout the rat brain

To validate psilocybin-induced acute changes in brain activity complementary to fMRI readouts, immunostaining of EGR1 was performed and six slices were selected according to the significant DC changes in cortical and subcortical regions like the cingulate cortex, prefrontal cortex, striatum, hippocampus, retrosplenial cortex, and some thalamic regions. Images of representative brain regions are shown in Figure 4. In our IF counting procedures, subregions showing significant differences in EGR1 expression were elaborately counted and illustrated in the same graphs. Psilocybin tended to increase EGR1 expression across the brain, with significant increases in the primary somatosensory cortex, insular cortex, striatum, nucleus accumbens, medial septum, preoptic area, amygdala, hypothalamus, parietal and temporal association cortex, auditory cortex, piriform cortex, hippocampus, visual cortex, dorsal subiculum, retrosplenial granular cortex, visual cortex, and ventral tegmental area (Figure 5). Furthermore, no decrease in EGR1 level was observed in our IF images.

**Figure 4:** Representative immunofluorescence images of increased EGR1 in different regions. **(A)** prelimbic region, PrL, **(B)** cingulate cortex, Cg, **(C)** retrosplenial granular cortex, RSG, **(D)** primary somatosensory cortex, upper lip, S1ULp, **(E)** primary auditory cortex, Au1, **(F)** primary visual cortex, monocular, V1M, **(G)** insular cortex, Ins, **(H)** caudate putamen (striatum), CPu, **(I)** filed CA1 of the hippocampus, CA1, **(J)** amygdala, Amy. Scale bars, 800 μm in yellow, 200 μm in white.

**Figure 5:** Increased EGR1 expression after psilocybin. Density of EGR1 positive neurons in different coronal sections (AP): **(A)** + 3.24 mm, **(B)** + 0.96 mm, **(C)** −0.24 mm, **(D)** −2.04 mm, **(E)** −3.84 mm, **(F)** −5.88 mm. The abbreviations of the IF brain regions were listed in Supplementary Table S2. Data are shown as mean ± SEM, multiple unpaired t test, compared with saline group, * *p* < 0.05, ** *p* < 0.01, *p* value ranging between 0.05 and 0.1 are directly annotated in the graphs, *n* = 3 per group.

## 4. Discussion

In this study, psilocybin-induced brain activity changes were investigated using BOLD fMRI and EGR1 IF techniques. DC analysis, ROI-wise FC analysis, and cingulate cortex-based FC analysis were performed to investigate psilocybin-induced brain changes from different perspectives, presenting a mixed pattern of brain activity and connectivity changes characterized by generally increased activities and FC in the cortical and striatal regions and decreased activity in several subcortical regions. Among them, the hub regions like the cingulate cortex may be the key regions psilocybin affected.

The article "Acute psilocybin increased cortical activities in rats" was retracted in 2026. Reasons: errors in the materials; unreliable results or conclusions.

Increased degree centrality was observed in the cortical and some subcortical areas, especially in prelimbic areas, cingulate cortex, striatum, and hippocampus. Decreased activity was observed in such subcortical areas such as the accumbens shell, some basal thalamic nuclei, and hypothalamic nuclei (Figure 1). In cortical regions, EGR1 expression was also widely activated, with significant increases in somatosensory, auditory, visual, and insular cortices (Figures 4, 5). Widely increased BOLD signals and EGR1 expression across different cortical regions suggested psilocybin may elicit a hyper-cortical state in rats. Consistently, a positron emission tomography (PET) study in healthy volunteers reported that acute psilocybin treatment induced a hypermetabolic state in most cortical regions reflected from the striking increase in prefrontal metabolic rate of glucose (Vollenweider et al., 1997). However, in contrast to the acute effects, another long-term study reported specifically decreased glutamate and N-acetylaspartate (NAA) levels in ACC of patients with major depressive 1 week after psilocybin treatment (Doss et al., 2021). These two studies imply that psilocybin may elicit different acute versus chronic effects, which deserves detailed investigation but is beyond the scope of this research. Congruent with human studies, consistent results that optogenetic stimulation of mPFC produced antidepressive effects and concurrently increased IEG EGR1 and FOS expression were observed in depression-phenotype susceptible mice, suggesting the neural activity in the hub regions as a determinant of antidepression responses (Covington et al., 2010).

Cingulate regions between humans and rodents bear both similarities and dissimilarities. In humans, the cingulate cortex is a significant hub region for association, cognitive flexibility, emotional processing, learning, and memory. And in rats, this hub region is also important for inter-hemispheric communication. With reference to anatomical structures, the cingulate cortex in rats is composed of Cg1 and Cg2 (Supplementary Figure S1B; Paxinos and Watson, 2007) and is homologous to ACC and the medial cingulate cortex (MCC) in humans (Vogt and Paxinos, 2014). And human PCC is cytoarchitecturally equivalent to rat retrosplenial cortex (RSC), which comprises both retrosplenial granular and dysgranular cortices (RSG/RSD) (Lu et al., 2012; Vogt and Paxinos, 2014). However, in the fMRI templates (Barrière et al., 2019) we used, the rat cingulate cortex was functionally divided into three subregions, Cg1/2/3, among which Cg1 and Cg2 were identified as the homolog of ACC in humans, and Cg3 of MCC in humans (Supplementary Figure S1A; Vogt and Paxinos, 2014).

The article "Acute psilocybin increased cortical activities in rats" was retracted in 2026. Reasons: errors in the materials; unreliable results or conclusions.

Our brain-wide FC analysis revealed mostly increased interconnection of Cg3 with other brain regions; interconnection of Cg1 and ventral striatum also changed significantly (Figure 2). Likewise, IF results showed that psilocybin increased EGR1 in cingulate regions, although not significantly (Figure 5). In consideration of the importance of cingulate cortex in depression-relieving effects of psilocybin, anatomical cingulate cortex-based (Supplementary Figure S1B) seed analysis was performed, showing its hyperconnectivity with wide cortical and some subcortical areas including the olfactory bulb, orbital frontal cortex, insular cortex, entorhinal cortex, visual cortex, retrosplenial cortex, striatum and hippocampal dentate gyrus, and hypoconnectivity with septum, piriform cortex, amygdala, inferior thalamic areas, and substantia nigra (Figure 3), which suggested the importance of the hub region in psilocybin-induced brain activity alterations. Similarly, patients with major depressive disorder (MDD) show decreased module allegiance matrix (MAM) value between ACC and different regions like the insular cortex, amygdala, precuneus, and thalamus, suggesting a lowered interconnection strength in depressive condition (Zheng et al., 2018), which was reversed after psilocybin administration, characterized by increased inter-regional FC, decreased brain modularity, and reduced hierarchical organization after the antidepressant treatment (Roseman et al., 2014; Carhart-Harris et al., 2017; Doss et al., 2021; Daws et al., 2022; Girn et al., 2022). This implies the pivotal role of the cingulate cortex in psilocybin-induced brain activity changes in both humans and rats.

Elevated EGR1 expression in both cortical and subcortical areas revealed a brain-wide ‘neural activation’ blueprint, although, in some regions, increased EGR1 were just trends but did not reach the statistically significant threshold. The two experiments showed convergent neural activation in many brain regions including the prefrontal, cingulate, sensory-related, insular, and retrosplenial cortex, hippocampus, and striatum, areas closely related to multiple sensory-processing, emotion, association, cognitive flexibility, and memory. The increased cortical activities, especially in PFC and the cingulate cortex, and increased interconnectivity of the cingulate cortex may be the mechanism through which psilocybin exerts potent psychoactive effects.

The article "Acute psilocybin increased cortical activities in rats" was retracted in 2026. Reasons: errors in the materials; unreliable results or conclusions.

Regardless of good coherence, however, there were still undesirable but predictable discrepancies between fMRI and IF outcomes, which necessitate detailed elucidation. For example, areas with positive BOLD signals are not absolutely consistent with those showing significantly increased EGR1 levels. In addition, decreased BOLD signals were observed in some thalamic and hypothalamic areas, whereas no reduction in EGR1 level was observed.

The principle of BOLD fMRI is important to understand the inconsistencies. All brain activities are energy-consumptive, including both excitatory and inhibitory processes. BOLD signals indirectly reflect the mass action of neuronal assembles from the hemodynamic changes induced by varied brain processes (Glover, 2011), known as neurovascular coupling, which is ambiguous in its nature (Buzsáki et al., 2007). In substantial cases, excitation consumes more energy than inhibition does (Buzsáki et al., 2007). But the relationships between BOLD signals and neural activities still remain not fully understood, especially when interpreting negative signals. From a perspective of excitation-inhibition balance, a positive fMRI signal in a brain region is usually associated with increased activity, which may result from 1) direct excitation activation, 2) proportional activation of both excitation and inhibition leading to unchanged local neural activity but increased metabolism, or 3) indirect excitation activation secondarily resulting from deactivation of inhibition, which causes net excitation in the conditions. However, given the complexity of hierarchical organization and multiplicity of circuits and microcircuits, a net inhibition in a certain brain region may generate either positive or negative BOLD signals in a circuit-dependent manner (Logothetis, 2008). For example, early shunting of an excitatory input may lead to decreased recurrent excitation, in which a clear negative BOLD signal occurs, but increased synaptic inhibition or early shunting of an output may result in a positive signal (see the review for detail (Logothetis, 2008)). It was reported that isoflurane enhanced inhibition of thalamic neurons in the ventrobasal thalamus via GABA_A_R-dependent, but in reticular thalamic nucleus (RTN) via GABA_A_R independent mechanisms (Ying et al., 2009), which may help to interpret the negative BOLD signals in basal thalamic nuclei in our fMRI readouts.

Apart from GABAergic inhibition enhancement (Fracasso et al., 2022), dopamine system activation is sufficient to elicit decreased striatal fMRI signals in rats via dopamine D_2_ receptor (D_2_R) stimulation (Shih et al., 2009; Hsu et al., 2014). A human PET study shows that psilocybin indirectly facilitates dopamine release through stimulation of 5-HT_1A_ and 5-HT_2A_ receptors (Vollenweider et al., 1999). And psilocybin produced increased FC of mouse brain between 5-HT-associated networks and decreased FC between dopamine-associated networks (Grandjean et al., 2021). In addition to the IF results that psilocybin elevated EGR1 levels in dopamine-related regions like VTA (Figure 5), we therefore speculate that psilocybin-induced negative subcortical BOLD signal may, at least partially, attribute to dopamine or GABA activation or a combination of them.

The article "Acute psilocybin increased cortical activities in rats" was retracted in 2026. Reasons: errors in the materials; unreliable results or conclusions.

A “bipartite” model theory was also proposed that brain serotonin mediates adaptive responses to adversity through respective 5-HT_1A_R signaling for stress modulation and 5-HT_2A_R signaling for adaptation (Carhart-Harris and Nutt, 2017). In this research, psilocybin-induced hyperactivity across cortical and some subcortical regions bore great similarity with the distribution of 5-HT_2A_ receptors, consistent with the spatially heterogeneous gene expression pattern of 5-HT_1A_R, 5-HT_2A_R receptors across primate and rodent brains (Burt et al., 2018; Preller et al., 2020; Grandjean et al., 2021), indicating the crucial role of the two receptors in psilocybin-induced brain activity alteration.

BOLD fMRI scanning detects the neurovascular coupling event and stimulation-induced cerebral blood flow (CBF) as an important factor worth considering. Besides, brain 5-HT plays a major vasoconstrictor role, increases in which, both directly and indirectly, leads to reduced CBF (Cohen et al., 1996). And several serotonin receptors are involved in the complicated vasculature effects, including 5-HT_1B_, 5-HT_1D_, and 5-HT_2A_ receptors, for which psilocin, the active metabolite of psilocybin, has high affinity, making the BOLD signals difficult to understand (Cohen et al., 1996; Elhusseiny and Hamel, 2001; Hamel, 2006; Lewis et al., 2017). However, a hemodynamic study in humans suggests that psilocybin decreases global CBF but bidirectionally modulates regional CBF with increments in the right frontal and temporal regions, bilateral fluctuation in the anterior insula, and decrements in the left parietal and occipital regions, amygdala, globus pallidus, insula, and thalamus, using pseudo continuous arterial spin labeling (pCASL) fMRI (Lewis et al., 2017), indirectly reflecting a hyper-frontal and hypo-subcortical pattern, corresponding to our fMRI readouts to some extent.

In view of the fact that anesthesia can influence neural activity, our experimental design, in which BOLD fMRI and EGR1 IF were performed simultaneously but using separate rats from the same batch, was based on the following considerations.

The article "Acute psilocybin increased cortical activities in rats" was retracted in 2026. Reasons: errors in the materials; unreliable results or conclusions.

Serotonergic neurons in the dorsal raphe nucleus (DRN) were reported to be inhibited following isoflurane anesthesia (Johansen et al., 2015; Yang et al., 2019), which could in turn influence the activities of brain-wide neurons expressing serotonin receptors (Mukaida et al., 2007) and even reconfigure the prefrontal neurotransmitter network composing of glutamate, GABA, dopamine, acetylcholine, adenosine, norepinephrine, histamine, and serotonin (Zhang et al., 2020). However, on account of the potential but great influence of mental stress induced by forced fixation and the common HTR effect (Supplementary Figure S2) produced by psilocybin and other hallucinogenic 5-HT_2A_ receptor agonists in awake rodents, fMRI scanning under an anesthetic state is an eclectic but necessary method for rodent neuroimaging.

General anesthesia also prevents activity-induced initiation of IEG *egr1* transcription, consequently resulting in reduced EGR1 levels, but does not stop ongoing *egr1* transcription and subsequently does not influence the expression of EGR1 (Bunting et al., 2015). More importantly, it was reported that isoflurane-elicited prolonged changes of protein expression in rats could persist for several days (Kalenka et al., 2010). Based on this, IF rats were kept unanesthetized rather than anesthetized until the transcardial perfusion operation to exclude the possibility that psilocybin-induced EGR1 changes might be blunted under post-isoflurane condition. IEGs are critical mediators of gene × environment interactions (Guzowski et al., 1999). As a result, EGR1 IF in this study may reflect co-effects of psilocybin and potentially environmental stimuli, which may contribute to additional differences between BOLD signals and IF results. But experiments with conscious animals can better reflect the real situation. Besides, each rat was well acclimatized to the experimental environments and every effort was made to minimize the confounding influence of any environmental factors during the operation.

Although this experimental design disabled the one-for-one comparison between fMRI readouts and IF EGR1 counts of each rat and may likely introduce additional factors (anesthetic state or the environment), the group-wide comparison also differentiated the affected brain regions as mentioned above.

Aisling Spain and her colleagues reported seemingly discrepant results that rats with a single dose of 2 mg/kg psilocin produced a negative signal in the cingulate and somatosensory cortex, but a positive signal in the hypothalamus and amygdala (Spain et al., 2015). Here, we try to give our explanation. In their research, a dose of 2 mg/kg psilocin was intravenously injected into rats, which may lead to a sharp rise in blood psilocin concentration. In contrast, 2 mg/kg psilocybin hydrochloride was intraperitoneally administered through a homemade injection device in our research. Therefore, the injected psilocybin was, at first, converted into psilocin. Then the bioactive psilocin could be absorbed into the circulation system (Eivindvik et al., 1989), which was likely to maintain a milder and more sustained concentration and to take more moderate effects. Furthermore, the relative potency of psilocin to psilocybin is identical to their molecular mass ratio (Wolbach et al., 1962), while psilocybin hydrochloride has a larger molecular mass than psilocin, indicating the dosage employed in this research was much lower than that in theirs (Spain et al., 2015).

The article "Acute psilocybin increased cortical activities in rats" was retracted in 2026. Reasons: errors in the materials; unreliable results or conclusions.

Our HTR results presented a bell-shaped HTR curve in a dose-dependent manner, and the 2 mg/kg psilocybin hydrochloride located on the descending phase could still significantly increase HTR bouts (Supplementary Figure S2A), which suggested different receptors may be involved in different phases. Psilocin has affinities for multiple serotonin receptors including 5-HT_1A_ and 5-HT_2A_ receptors. The two may constitute a “bipartite” model for serotonergic modulation, which was hypothesized to refer to passive and active coping, respectively (Carhart-Harris and Nutt, 2017). And the inhibitory role of the 5-HT_1A_ receptor in psilocybin- or psilocin-induced effects, including HTR, was reported (Shahar et al., 2022); therefore, the descending phase may be on account of the inhibitory effects of 5-HT_1A_ receptor activation (Darmani et al., 1990). The 2 mg/kg psilocin in their research may, therefore, present stronger inhibitory effects. Given this, we speculate psilocybin and psilocin may have biphasic effects on fMRI signals in a dose-dependent manner, which may explain the differences between the two studies. Furthermore, in Aisling Spain’s research, surgeries were performed and stimulant paradigms were carried out, which may compromise the states of rats and introduce confounding factors.

There still exist some technical considerations and limitations deserving exploration. Brain activity and connectivity is almost bidirectional, characterized by simultaneously increased and decreased BOLD signals detected in varied brain regions, while only unilaterally increased EGR1 expressions, though not significantly in some regions, were observed. EGR1 is widely expressed cross-brain and the immunostained EGR1 is the cumulative expression of all cell types in certain regions, but whether it has a cell-type specific expressing pattern still remains unclear, which may perplex our understanding of excitation or inhibition of specific regions where the constituent neuron types are varied. In future research, bilaterally modulated biomarkers or a combination of different cell-type specific ones may help to understand the bidirectional fMRI signals and further elucidate specific cell types involved in these neural activities.

The article "Acute psilocybin increased cortical activities in rats" was retracted in 2026. Reasons: errors in the materials; unreliable results or conclusions.

Activation of 5-HT_1A_ and 5-HT_2C_ receptors endows serotonergic system arousal-promoting effect, whereas receptors like 5-HT_1B_, 5-HT_2A_, 5-HT_3_, 5-HT_6_ and 5-HT_7_ have little effects (Li et al., 2021). How psilocybin influences the depth of anesthesia remains unclear. And hallucinogens targeting 5-HT_2A_ receptors induce HTR in both mice and rats (Halberstadt et al., 2020), circumventing the fMRI scanning under awake condition. There may be a critical conscious-anesthetic state where HTR is totally inhibited and the brain activities closely resemble that in conscious state, which will be of particular significance for fMRI research into hallucinogens in rodents.

In this fMRI study, predefined referential templates (Barrière et al., 2019), different to the stereotaxic atlas in IF experiments, were used to parcellate the fMRI data, in which a probability of mismatch or localization errors may occur especially in the outside edge of the two atlases due to architectural and volumetric differences between each individual. The margins of BOLD signal clusters may also vary, depending on the methodologies adopted (Guzowski et al., 1999). The fMRI templates (Barrière et al., 2019) and anatomical rat atlas (Paxinos and Watson, 2007) do not categorically match each other; some mismatch may occur especially around outside edges and in certain small nuclei. Therefore, higher resolution fMRI may be important for more accurate location of affected brain regions (Romanov et al., 2019) and more mutually-matched atlases are needed for comparison.

## 5. Conclusion

Despite technical limitations, it can be concluded that psilocybin produces hyperactivity and hyperconnectivity in a range of cortical regions and especially in the cingulate cortex in rats, indicating the “hub regions” such as mPFC, cingulate cortex, and retrosplenial cortex, play a key role in psilocybin-induced brain activity and connectivity changes. And our first combination of BOLD fMRI and IF EGR1 provides another way to better understand the complicated effects of psilocybin in rats.

## Data availability statement

The original contributions presented in the study are included in the article/Supplementary material, further inquiries can be directed to the corresponding authors.

## Ethics statement

The animal study was reviewed and approved by Ethics Committee and Institutional Animal Care and Use Committee of Beijing Institute of Pharmacology and Toxicology.

The article "Acute psilocybin increased cortical activities in rats" was retracted in 2026. Reasons: errors in the materials; unreliable results or conclusions.

## Author contributions

JL, HY, and RS contributed to conception and design of the research. JL performed the main experiments and wrote the first draft of the manuscript. YW, JW, KX and DZ participated in part of the experiments. JL, YW, JW, and AC participated in data processing and analysis. AC, HY, and RS revised the manuscript. All authors contributed to the article and approved the submitted version.

## Funding

This study was sponsored by the fund Logistics Research Project (BWS17J022).

## Conflict of interest

The authors declare that the research was conducted in the absence of any commercial or financial relationships that could be construed as a potential conflict of interest.

The handling editor SL and reviewer BN declared a past co-authorship with the authors JW and AC.

## Publisher’s note

All claims expressed in this article are solely those of the authors and do not necessarily represent those of their affiliated organizations, or those of the publisher, the editors and the reviewers. Any product that may be evaluated in this article, or claim that may be made by its manufacturer, is not guaranteed or endorsed by the publisher.

## Supplementary material

The Supplementary material for this article can be found online at: https://www.frontiersin.org/articles/10.3389/fnins.2023.1168911/full#supplementary-material

## Footnotes

^1^ https://afni.nimh.nih.gov

^2^ https://fsl.fmrib.ox.ac.uk/fsl/fslwiki/

^3^ https://github.com/ANTsX/ANTs

^4^ https://people.cas.sc.edu/rorden/mricro/Bru2anz
